# Cognitive workload evaluation of landmarks and routes using virtual reality

**DOI:** 10.1371/journal.pone.0268399

**Published:** 2022-05-17

**Authors:** Usman Alhaji Abdurrahman, Lirong Zheng, Shih-Ching Yeh

**Affiliations:** 1 School of Information Science and Technology, Fudan University, Yangpu District, Shanghai, China; 2 Department of Computer Science, Yusuf Maitama Sule University, City Campus, Kano, Nigeria; Al-Balqa Applied University Prince Abdullah bin Ghazi Faculty of Information Technology, JORDAN

## Abstract

Investigating whether landmarks and routes affect navigational efficiency and learning transfer in traffic is essential. In this study, a virtual reality-based driving system was employed to determine the effects of landmarks and routes on human neurocognitive behavior. The participants made four (4) journeys to predetermined destinations. They were provided with different landmarks and routes to aid in reaching their respective destinations. We considered two (2) groups and conducted two (2) sessions per group in this study. Each group had sufficient and insufficient landmarks. We hypothesized that using insufficient landmarks would elicit an increase in psychophysiological activation, such as increased heart rate, eye gaze, and pupil size, which would cause participants to make more errors. Moreover, easy and difficult routes elicited different cognitive workloads. Thus, a high cognitive load would negatively affect the participants when trying to apply the knowledge acquired at the beginning of the exercise. In addition, the navigational efficiency of routes with sufficient landmarks was remarkably higher than that of routes with insufficient landmarks. We evaluated the effects of landmarks and routes by assessing the recorded information of the drivers’ pupil size, heart rate, and driving performance data. An analytical strategy, several machine learning algorithms, and data fusion methods have been employed to measure the neurocognitive load of each participant for user classification. The results showed that insufficient landmarks and difficult routes increased pupil size and heart rate, which caused the participants to make more errors. The results also indicated that easy routes with sufficient landmarks were deemed more efficient for navigation, where users’ cognitive loads were much lower than those with insufficient landmarks and difficult routes. The high cognitive workload hindered the participants when trying to apply the knowledge acquired at the beginning of the exercise. Meanwhile, the data fusion method achieved higher accuracy than the other classification methods. The results of this study will help improve the use of landmarks and design of driving routes, as well as paving the way to analyze traffic safety using the drivers’ cognition and performance data.

## 1. Introduction

One of people’s daily routines is navigating from one route to another. This includes moving from home to work, from a particular shop to another, and from offices to visiting friends [1]. While navigating, people tend to make sequential decisions, such as going straight, turning left, or turning right; this is called route knowledge [2]. Apart from route knowledge, other essential information is required for effective navigation. Information such as metrics is acquired from sensory sources, while features (e.g., landmarks) are perceived visually [3]. It was discovered that, in the course of route-finding, people tend to make one error per week on average, with 49% of those errors occurring when people turn in the wrong direction [4]. Metrics and feature information are needed to reduce the number of mistakes during navigation, as they play a vital role in enriching people’s knowledge. Feature information, such as landmarks, affects our ability to navigate effectively, as they provide positional and orientation information. Landmarks reflect spatial information of natural objects, reduce subjects’ cognitive loads, and increase their navigational efficiency [5]. Successful wayfinding requires accurate integration and memory of landmarks in their spatial relations [6].

Thus, landmarks may be categorized into local and global [7–9]. According to Waller et al. [10], local landmarks can be associative or beacons; associative landmarks indicate a decision point’s position, while beacon landmarks indicate both the position and how one should turn. Previous studies showed that environmental landmarks reduce participants’ mistakes when traversing a route. The landmarks help participants to apply the knowledge acquired while traversing a route from one direction when returning to the other [11].

In the current study, participants used landmarks to locate their respective destinations. Landmarks can be any distinctive point used for navigation, such as buildings, intersections, and streets [6, 12, 13]. In this study, locations such as a basketball court, a McDonald’s, a convenience store, a gas station, a post office, a church, and a Walmart were used as the primary source of landmarks. We will refer to these locations as landmarks in the subsequent sections. Therefore, we hypothesized that sufficient landmarks would reduce the overall number of mistakes that participants make during a navigational exercise.

One of the targets of this study was the measurement of navigational efficiency, which is the time required by the participants to complete an assigned task. In this study, participants were given the task of recognizing routes based on landmarks to reach their destination. The navigational efficiency was determined by analyzing the recorded data of the participants using driving performance metrics. Consequently, we hypothesized that the navigational efficiency of routes with sufficient landmarks would be remarkably higher than that of routes with insufficient landmarks.

Moreover, complex routes affect drivers because they have to process more information, which in turn increases their driving cognitive workload. As defined by Senders [14], the workload is a measure of effort dissipated by a human operator while performing a task, regardless of the performance of the task itself. When workload levels are low, the performance is also low because of inattention and missed information. As the workload increases, the level of performance increases as well up to a maximum level. This maximum performance represents the optimal workload level for a given task. An additional mental workload leads to an abrupt decrease in performance because of the extra amount of information to be processed, resulting in a high cognitive workload [15]. According to Sweller [16], the cognitive workload is the total amount of cognitive resources needed to process information in cognitive activities. The cognitive workload is characterized by psychophysiological changes (e.g., alterations in heart rate and skin conductance, and behavioral approach or avoidance). It involves several subcomponents occurring in frontal subcortical circuits [17, 18]. Therefore, we hypothesized that the easy and difficult routes used in our study would elicit different cognitive workloads. In addition, a high cognitive load would negatively affect the participants applying the knowledge acquired at the beginning of the exercise.

Several studies investigated the measurement of driving behavior using different psychophysiological parameters [19–22]. Pupil size is well known to respond rapidly to changes in brightness in the visual field and has been used to measure the cognitive load while performing an assigned task [19, 22]. Research shows that heart rate increases when a participant is subjected to more challenging conditions [23–26]. According to Brookhuis et al. [27], an increase in task demand, such as entering a traffic circle, increases the heart rate, which in turn decreases with the demand, e.g., driving on a two-lane highway. An increase in respiratory rate has been often related to an increase in cognitive demand [26, 28, 29]. Another essential metric that has been found to increase as the cognitive workload increases is skin conductance [21]. Electroencephalogram (EEG) signals are sensitive and reliable for cognitive load measurement [30, 31]. Thus, in this study, heart rate and pupil size were used to measure the cognitive workload of the participants during the navigation exercise.

The application of previously acquired knowledge and skills in new learning or problem-solving situations is termed as transfer of learning [32]. According to Perkins et al. [33], transfer of learning is said to occur when learning in one context enhances (positive transfer) or undermines (negative transfer) a related performance in another context. It expresses the ability to transfer what was learned from one context or situation to another [34]. Some previous studies argued that transfer is only possible when the original and the new learning situations are the same or very similar; this is termed as a near-transfer. Other researchers achieved transfer across different learning situations, termed as far-transfer [35]. However, the degree of transfer increases as the similarity of the elements increases. Thus, we used similar elements in our study to simplify the process of learning transfer.

Virtual reality (VR) technology was used to achieve the stated objectives. VR technology can create immersive and realistic interactive environments for behavioral learning. Besides, VR technology provides individualized treatment, accurate control of complex stimuli, and a structured and safe learning environment [36, 37]. Therefore, we employed a VR-based driving system to investigate the effects of landmarks and routes on navigational efficiency and transfer of learning.

The remaining sections of this paper are organized as follows: Section 2 presents the methods employed and the experiments conducted in this work. Section 3 presents the results obtained from the experiments. Section 4 gives a thorough analysis of the presented results. Section 5 concludes the paper.

## 2. Methods and experiments

### 2.1 Hypotheses

This study aimed to evaluate the effects of different landmarks and routes on navigational efficiency using a VR-based driving system. Psychophysiological metrics such as heart rate, eye gaze, pupil size, and driving performance features were used to assess the cognitive load experienced by the participants. Thus, we hypothesized the following points:

1. The use of insufficient landmarks would elicit an increase in psychophysiological activation, such as increased heart rate, eye gaze, and pupil size.
2. An increase in psychophysiological activation would cause the participants to commit more errors.
3. The navigational efficiency of routes with sufficient landmarks is remarkably higher than that of routes with insufficient landmarks.
4. The easy and difficult routes would elicit different cognitive workloads. In addition, a high cognitive load would negatively affect the participants applying the knowledge acquired at the beginning of the exercise.

### 2.2 Participants

Seventy-nine (79) undergraduates, distributed as 36 males and 43 females, from Fudan University participated in the experiment. The participants age between 18 and 24 years old (Age: M = 19.27; SD = 2.31) and were recruited through in-house advertisement. No significant differences were found in terms of age, education, or gender. The participants were divided into two (2) groups; group X and group Y. Group X had 39 participants (18 males and 21 females), and group Y had 40 participants (18 males and 22 females). All volunteers had normal eyesight and no real-life driving experience. Before conducting the experiment, the participants filled out a consent form, and approval was granted by the university. All participants received a reward after the experiment. The recorded data were analyzed, and they are reported below.

### 2.3 Experimental materials

The experiments were conducted at Fudan University. The VR driving system used in this study is illustrated in Fig 1. The materials used include Vive Pro Eye for tracking eye data [38] and a Logitech G27 steering-wheel controller for controlling the virtual agent vehicle in the driving environment. An Autodesk Maya [39] and Esri CityEngine [40] were used to design landmarks, traffic lights, routes, intersections, cars, and buildings, while Unity3D [41] was used to develop the game platform. The driving routes consisted of city roadways that comprised long straightaways, several turns, intersections, and landmarks (such as a basketball court, a McDonald’s, a convenience store, a gas station, a post office, a church, and a Walmart). Two difficulty levels were developed for the VR-based driving system, with each level comprising two driving assignments.

**Fig 1:** VR driving system. A participant driving in the virtual system (left) and a snapshot containing the ego vehicle, sample of the driving route, intersection, and landmark within the virtual system (right).

The data capture module recorded the participant’s information while driving. A Vive Pro eye tracker recorded the eye-gaze data (including the pupil size and gaze origin) at 50 Hz. A heartbeat recording device designed in our laboratory was used to track the subject’s heart rate at 500 Hz while driving in the virtual environment.

### 2.4 Experimental procedure

All participants submitted their informed consent forms before the commencement of the experiments. The experiments were conducted according to relevant guidelines and regulations. As stated earlier, there were two (2) groups. Each group had two (2) sessions in the study: group X1 (sufficient landmarks and easy routes), group X2 (insufficient landmarks and easy routes), group Y1 (sufficient landmarks and difficult routes), and group Y2 (insufficient landmarks and difficult routes). The two sessions per group presented the same difficulty; however, the number of landmarks varied. Group X1 had seven landmarks, group X2 had three landmarks, group Y1 had seven landmarks, and group Y2 had five landmarks. The easy routes had three turns, intersections, and three traffic lights, while the difficult routes had five turns, intersections, and five traffic lights. Each participant completed two (2) sessions of the assigned group (either X1 and X2, or Y1 and Y2).

Baseline data were recorded prior to the experiments. Then, a video tutorial was given to the participants to introduce them to the routes they were going to follow, as well as the landmarks, intersections, and traffic lights they were going to see, to help them complete the given task. This video was played only once, and the participants were asked to memorize all the landmarks along the routes. The staff then set up the eye-tracking and heartbeat sensors on the subject’s body and ensured that all signals were properly recorded and the devices operated perfectly. The subjects were then asked to carry out the pre-selected driving assignment based on the video tutorial they had just watched.

The subjects used the landmarks along the routes to locate the right turns to take them to their various destinations. Thus, whenever a subject made a wrong turn, they were dragged to the starting point to re-watch the video tutorial and start driving all over again. The tutorial sessions were included to assess the system and improve the subject’s driving performance. However, we did not consider the performance of these sessions in data analysis.

### 2.5 Experimental design and data collection

This study employed a VR-based driving system to determine the effects of landmarks and routes on navigational efficiency and learning transfer. We chose the between-group design of 2 (landmarks: sufficient landmarks and insufficient landmarks) x 2 (routes: difficult routes and easy routes). The participants in each group completed two (2) sessions of the four tests (either X1 and X2, or Y1 and Y2).

All physiological measures such as pupil size and heart rate, and the driving performance data were generated from each session during the experiment. Data for all 79 subjects were extracted for analysis. To enhance the credibility and robustness of the results, all the generated data were preprocessed to remove the undesired parts. The median value method was used to reduce the noise level of the eye gaze data. Pupil size data were extracted from the eye gaze data. We extracted the following ten features from the eye gaze data, motivated by previous studies [19, 20]: fixation rate; blink rate; mean (M) and standard deviation (SD) of blink duration; M and SD of fixation duration; M and SD of pupil size; and M and SD of saccade duration. Similarly, M and SD were also extracted from the heart rate data.

Data related to the participants’ task performance were also generated. The performance features indicate how well a participant completed the assigned task; some examples of these features are the task completion time, wrong turns, and collision counts. The performance features used in this study and their meanings are listed in Table 1. We extracted six features: M and SD of task completion time, M and SD of wrong counts, and M and SD of barricade counts. The extracted data were used as the input vectors for the data fusion method.

**Table 1:** Performance features and their meaning.

Performance Feature	Meaning
Task completion time	Task completion time (in seconds)
Wrong turns	Total number of wrong turns
Collision counts	Total number of collisions on the edge of the road

#### 2.5.1 Navigational efficiency determination

One of the primary objectives of this study was to investigate the effects of landmarks and routes on navigational efficiency. After the participants completed their assigned task successfully, the total time spent (task completion time) in completing the task and the number of mistakes (wrong turns) were recorded in terms of driving performance metrics. The recorded data were used to determine the navigational efficiency of the assigned task.

#### 2.5.2 Learning transfer determination

We also investigated whether landmarks and routes influence learning transfer. This was achieved by evaluating the differences in psychophysiological response patterns associated with driving along the routes (easy and difficult) and landmarks (sufficient and insufficient). All psychophysiological metrics (such as drivers’ pupil size and heart rate) and performance measures were recorded simultaneously throughout the experiment. All these data were used to determine the subjects’ cognitive load, which, by extension, helped assess its effect on learning transfer.

### 2.6 Data fusion methods

The extracted features from different modalities were input into the classifiers to assess the participants’ cognitive workload. Five (5) popular classifiers (Table 5) were used to classify the cognitive workload in this study: a Support Vector Machine (SVM), an Artificial Neural Network (ANN), Naïve Bayes (NB), K-Nearest Neighbor (KNN), and a Decision Tree (DT). Three-level approaches for data fusion were used, namely feature-level fusion, decision-level fusion, and hybrid-level fusion. The structures of the data fusion methods used to fuse multimodal information are shown in Fig 2.

**Fig 2:** The structures of the data fusion methods. A feature-level fusion (a), a decision-level fusion (b), and a hybrid-level fusion (c).

Fig 2A depicts feature-level fusion. The extracted features from the eye gaze, heart rate, and driving performance were input into the preprocessing module. The features were normalized there, and their dimensions were reduced using principal component analysis. The cognitive load was determined from the preprocessed data.

In decision-level fusion (Fig 2B), the extracted features from each modality were preprocessed separately and then input into different classifiers. These classifiers then output a cognitive load as a sub-decision (S_n_).

Finally, the fusion module added up these sub-decisions with weights (w) and computed the final cognitive load (CL_final_) according to the following expression:

$${CL}_{final}=w_{1}S_{1}+w_{2}S_{2}+w_{3}S_{3}+w_{4}S_{4}$$ (1)

Fig 2C depicts the hybrid-level fusion used in this study. It combines both feature-level and decision-level fusions. Heart rate and performance features were preprocessed through hybrid-level fusion to obtain a sub-decision. The remaining features (pupil size and eye gaze) were preprocessed separately, and additional decisions were obtained. The final sub-decision was obtained by adding all the sub-decisions with weights.

## 3. Results

This study aimed to investigate the effects of landmarks and routes on navigational efficiency and learning transfer using a VR-based driving system. There were 39 data points for group X1 (easy routes and sufficient landmarks) and X2 (easy routes and insufficient landmarks), and 40 data points for group Y1 (difficult routes and sufficient landmarks) and Y2 (difficult routes and insufficient landmarks), resulting in a total of 79 data points. Statistical and data fusion methods were used to analyze the data.

### 3.1 Statistical method

A t-test method was employed to assess the influence of landmarks and routes on cognitive load. The assessments were performed as follows:

#### 3.1.1 Assessment of spatial cognitive load

Participants’ cognitive loads were examined using recorded psychophysiological responses and driving performance features. The following responses were obtained.

**a**. **Response of psychophysiological measures with cognitive load**

A t-test method was employed for comparison. The heart-rate results show that group X using sufficient landmarks was significantly different from group Y using insufficient landmarks (t = -230.10, p = 1.89E-26). The heart rate of group Y (M = 76.2, SD = 10.1) was significantly higher than that of group X (M = 74.3, SD = 6.3). In addition, the heart rate of group X1 was significantly higher than that of group X2 (t = -147.65, p = 1.34E-14), and the heart rate of group X2 (M = 74.3, SD = 8.1) was significantly higher than that of group X1 (M = 73.2, SD = 4.3). Similarly, the heart rate of group Y1 was significantly different from that of Y2 (t = -158.32, p = 1.45E-16), and the heart rate of group Y2 (M = 76.8, SD = 9.4) was significantly higher than that of group Y1 (M = 75.1, SD = 7.6).

Furthermore, the results of the pupil size show that group X using sufficient landmarks was significantly different from group Y using insufficient landmarks (t = -19.49, p = 4.56E-13). The pupil size of group Y (M = 5.4, SD = 0.71) was significantly larger than that of group X (M = 4.3, SD = 0.64). Additionally, the pupil size of group X1 was significantly larger than that of group X2 (t = -17.20, p = 3.7E-12), and the pupil size of group X2 (M = 4.5, SD = 0.3) was significantly larger than that of group X1 (M = 3.9, SD = 0.7). Similarly, the pupil size of group Y1 was significantly different from that of group Y2 (t = -17.53, p = 4.8E-13), and the pupil size of Y2 (M = 5.4, SD = 0.71) was significantly larger than that of group Y1 (M = 4.9, SD = 0.31).

The results obtained from all the groups were associated with the nature of the routes and insufficient use of landmarks.

**b**. **Response of driving performance features with cognitive load**

Similar to psychophysiological measures, the results of driving performance measures (Table 2) show a significant difference between groups X and Y using the t-test method (t = 9.63, p = 2.3E-21). Likewise, the performance measures of group X1 were significantly different from those of group X2 (t = 6.41, p = 1.9E- 18), and the performance measures of group Y1 were significantly different from those of group Y2 (t = 7.32, p = 2.0E-19). As shown in Table 2, the performance features of participants who drove the difficult routes with insufficient landmarks were significantly higher than those who drove easy routes and sufficient landmarks.

**Table 2:** Driving performance features.

Performance Feature	Group			
	X1	X2	Y1	Y2
Completion time	203.13	250.34	289.37	347.85
Wrong turns	0.24	0.32	0.54	0.98
Barricade counts	0.25	0.36	0.58	0.95

Moreover, as hypothesized, participants who drove the difficult routes with insufficient landmarks made more mistakes than their counterparts who drove easy routes (Table 2). Cognitive workload significantly differed between difficult and easy routes regarding performance features (t = 5.54, p = 0.001), leading to a significant interaction between the two groups.

**c**. **Assessment of navigational efficiency**

Previous studies focused on the task completion time regarding navigational efficiency and cognitive workload. Task completion time is an essential indicator of the cognitive workload and plays a vital role in practical applications owing to its significant effect on learning transfer. A higher task completion time means that a participant had to use more mental capacity to identify the right way to follow, resulting in a more significant workload.

The navigational efficiency assessment can be obtained by analyzing the task completion time (as shown in Table 3) and observing whether intergroup differences exist owing to different landmarks and routes. The two-sample t-test method was used for intergroup comparison. The results show that the task completion time of group X1 was significantly different from that of group X2 (t = -90.83, p = 5.16E-12), and the task completion time of group X2 using insufficient landmarks (M = 250.34, SD = 42.05) was significantly higher than that of group X1 using sufficient landmarks (M = 203.13, SD = 22.48). Likewise, the task completion time of group Y1 was significantly different from that of group Y2 (t = -97.47, p = 7.10E-13). The task completion time of group Y2 using insufficient landmarks (M = 347.85, SD = 35.13) was significantly higher than that of group Y1 using sufficient landmarks (M = 289.37, SD = 32.54). The relationship between difficulty level and mean of the task completion time can be viewed in Fig 3.

**Fig 3:** Relationship between difficulty level and mean task completion time. Participants spent much time completing the task as the task difficulty level increased.

**Table 3:** Task completion time.

Level	Group	M	SD	t	p
Sufficient Landmarks	X1	203.13	22.48	-90.83	5.16E-12
Insufficient Landmarks	X2	250.34	42.05		
Sufficient Landmarks	Y1	289.37	32.54	-97.47	7.10E-13
Insufficient Landmarks	Y2	347.85	35.13		

Note: M = mean; SD = standard deviation; *t* = inferential statistic; *p* is the probability of obtaining test results.

**d**. **Effects of landmarks and routes on gender**

The use of insufficient landmarks and difficult routes influenced the participants according to their gender. The experimental results show that female participants generally drove slower than their male counterparts. This resulted in female participants spending much time to complete the exercise owing to the extra cognitive load. Moreover, the mean change applied to cognitive load and task completion time reveal the degree of these effects. As shown in Table 4, the mean change (ΔM_1_) in sufficient landmarks for females (ΔM_1_ = 142.70) was more significant than that for males (ΔM_1_ = 112.29). This indicates that insufficient landmarks influenced female participants more than their male counterparts, as shown in Fig 4.

**Fig 4:** Mean task completion time. Mean sufficient and mean difficulty.

**Table 4:** Task completion mean.

Source	Gender	Mean Sufficient Landmarks	Mean Insufficient Landmarks	ΔM_1_	Mean Easy Routes	Mean Difficult Routes	ΔM_2_
Task Completion Time	Male	194.13	306.42	112.29	189.34	324.53	135.19
	Female	207.25	349.95	142.70	210.32	343.54	133.22

Additionally, the mean change in difficult routes for males (mean difficulty) (ΔM_2_ = 135.19) was barely different from that for females (ΔM_2_ = 133.22). This indicates that the effect of difficult routes on navigational efficiency is similar for both sexes, as shown in Fig 4.

### 3.2 Data fusion method

#### 3.2.1 Feature-level fusion

Table 5 lists the single-modality classifiers used in this study. The accuracies of feature-level fusion versus single-modality algorithms are presented in Table 6. The feature-level fusion achieved the highest accuracy, 93.21%, compared to the single-modality algorithms. The best accuracy in heart rate was obtained from the KNN algorithm, while that of eye gaze, pupil size, and performance was obtained from the SVM algorithm.

**Table 5:** Single-modality classifiers.

Classifier Index	Algorithm	Parameters
1	SVM	Linear SVM
2		Quadratic SVM
3		Cubic SVM
4		Sigmoid SVM
5		Gaussian SVM
6		Polynomial SVM
7	KNN	Fine KNN
8		Medium KNN
9		Coarse KNN
10		Cosine KNN
11		Cubic KNN
12		Weighted KNN
13	ANN	Levenberg–Marquardt algorithm with 10 hidden neurons
14		Conjugate Gradient Backpropagation and with 10 hidden neurons
15		RPROP algorithm and with 10 hidden neurons
16		Gradient Descent with momentum and with 10 hidden neurons
17		Gradient Descent and with 10 hidden neurons
18	NB	Gaussian
19		Multinomial
20		Bernoulli
21	DT	Complex tree
22		Medium tree
23		Simple tree

**Table 6:** Feature-level fusion vs. single-modality classifiers (%).

Classifier Index	Pupil Size	Heart Rate	Eye Gaze	Performance	Feature Fusion
1	90.87	82.67	81.23	87.45	87.13
2	89.98	83.56	82.53	85.76	90.43
3	86.53	86.89	85.89	**89.67**	89.98
4	81.67	88.79	86.87	79.54	91.09
5	**91.67**	87.89	79.98	78.98	89.43
6	89.93	86.76	**89.73**	87.87	90.12
7	83.45	90.54	82.64	86.79	87.56
8	90.46	83.56	80.42	78.61	88.65
9	87.56	76.43	79.31	80.31	85.78
10	88.86	**90.78**	83.76	83.65	89.97
11	83.28	89.34	88.93	84.46	91.44
12	84.17	90.23	69.79	87.95	90.54
13	79.56	87.21	85.61	86.74	**93.21**
14	90.11	85.75	81.56	83.86	91.46
15	86.76	79.84	78.72	73.56	89.56
16	87.34	72.31	82.86	74.63	91.96
17	81.75	69.52	86.75	81.54	90.29
18	82.54	79.89	78.54	80.52	89.43
19	81.23	82.86	75.38	69.98	84.34
20	76.54	78.51	81.29	86.56	76.43
21	80.35	81.02	79.69	75.43	78.42
22	68.74	64.57	81.00	76.94	77.42
23	80.02	79.99	76.67	80.23	81.03
Average	84.49	82.56	81.70	81.78	87.64

#### 3.2.2 Decision-level fusion and hybrid-level fusion

All the classifiers for each modality were applied to decision-level fusion to obtain the sub-decision. Additionally, different combinations of weights were tested for every sub-decision. The best accuracy for the decision-level fusion, 91.45%, was obtained from the KNN algorithm.

The accuracy obtained from hybrid-level fusion was 95.34% higher than that of feature-level and decision-level fusions. This accuracy was achieved when pupil-size and eye-gaze features were combined for sub-decision one with the SVM algorithm, heart rate for sub-decision two with the KNN algorithm, and performance for sub-decision three with the ANN algorithm.

## 4. Discussion

The results just presented show that the use of landmarks (sufficient landmarks, insufficient landmarks) and routes (easy routes, difficult routes) affects the navigational efficiency and transfer of learning; however, the impact of these effects differs. This section thoroughly analyzes the results presented in the previous section.

### 4.1 Effect of landmarks on driving workloads

We hypothesized that sufficient landmarks would reduce the overall number of mistakes that participants make during navigational exercise. Sufficient landmarks reduced the participants’ number of mistakes from both easy and difficult routes. This can be concluded from the results in Table 2 concerning the response of driving performance features with cognitive load. This finding aligns with a previous study in which participants learned a route in one direction [42]. In addition, according to Ruddle [43], landmarks primarily facilitate traveling between specific places instead of assisting in learning the overall layout of a space. These landmarks provided positional information, which helped address the participants’ most common mistake: going straight instead of turning left or right.

Moreover, we hypothesized that the navigational efficiency of routes with sufficient landmarks would be significantly higher than that of routes with insufficient landmarks. This hypothesis was also supported by the results obtained regarding task completion time for all groups. In addition, these results are supported by previous studies [5, 11, 44]. The results show that the task completion times of groups X2 and Y2 was significantly higher than those of groups X1 and Y1, respectively. This happened because the participants required more cognitive resources (i.e., high cognitive load) in searching for the right routes to follow to reach the destination. Consequently, this negatively affected the participants in applying the knowledge acquired at the beginning of the exercise.

### 4.2 Effect of workloads on psychophysiological metrics

One of our primary analyses in this study was to evaluate the differences in psychophysiological response regarding navigation on easy routes using sufficient landmarks versus insufficient landmarks, and on difficult routes using sufficient landmarks versus insufficient landmarks. As anticipated, navigation using insufficient landmarks elicited increased psychophysiological activation in terms of, for instance, pupil size and heart rate. An increase in cognitive workload was related to the conditions of a cognitively challenging task (searching for the right turn owing to insufficient landmarks and difficult routes), which led to an increase in the response level.

The results obtained for the pupil size are supported by several findings, as indicated in [21, 45, 46]. According to Kahneman et al. [47], pupillary diameter increases as the amount of information loaded into working memory increases. In an experiment conducted by Querino et al. [45], the pupillary diameter was used to distinguish the cognitive effort between automated and controlled cognitive processing during the so-called five digits test (FDT) as the task progressed. The results show that, compared to a control task, the FDT required higher cognitive effort for each consecutive part, and the first half of every aspect of the FDT induced more size than the second.

Similarly, several previous studies also support our findings [48, 49]. According to Soroosh et al. [49], an increase in perceived cognitive workload appears to increase the sympathetic and parasympathetic components of the autonomic nervous system. Verway et al. [50] tested participants through cognitive tasks with respect to a control task in which no additional cognitive task was carried out while driving. The results show decreased heart rate variability and increased heart rate (decreased IBIs) when performing the cognitive tasks.

### 4.3 Effect of workloads on driving performance

In this study, we considered and investigated the task completion time, wrong turns, and collision counts for driving performance. These parameters were quantified and measured under different cognitive workloads, and the participants’ driving performance was assessed. Concerning the task completion time, participants in groups X2 and Y2 required more time to reach the destination than their counterparts in groups X1 and Y1. This happened because of the additional time needed by the participants to search for the right direction to reach the destination. This extra time also led to an increase in the cognitive workload of the participants, thereby hindering the transfer of learning. Our results are consistent with those of Fan H. et al. [5]. The navigational task-finishing time of the group using the full-landmark map was significantly higher than that of the group using the key-landmark map.

The wrong turns and collision counts were also higher in groups X2 and Y2 than in groups X1 and Y1 for the same reasons. The cognitively challenging task of searching for the right turn using insufficient landmarks was tedious, especially on difficult routes. This added more information to the participants’ working memory, which required more cognitive resources to process them. This result is in line with previous research conducted by Lyu et al. [51], in which the speed maintenance and lane deviations were significantly different under different levels of cognitive workload.

### 4.4 Effect of psychophysiological metrics and driving performance on gender

According to Underwood G. et al. [52], the cognitive workload is higher for novice drivers than for skilled drivers, as novice drivers need to pay much attention while driving. Therefore, only novice drivers were recruited for the experiments in this study. As shown in the results, insufficient landmarks and difficult routes presented a gender bias. The female participants paid more attention to the landmarks and drove slower than their male counterparts. Thus, they made more mistakes (higher wrong turns and collision counts) while driving. Moreover, female participants had higher task completion times than their male counterparts [19, 51].

### 4.5 Multimodal data fusion

For the single-modality classification, the best accuracy in heart rate (90.78%) was obtained from the KNN algorithm, while that of eye gaze (89.73%), pupil size (91.67%), and performance (89.67%) was obtained from the SVM algorithm. These results were consistent with the findings of Alzubi et al. [53]. In their study, an SVM combined with Harris Hawks optimization (HHO) for Android malware detection was proposed. It was observed that the proposed approach outperformed the baseline approaches on most datasets and measures.

It was verified that feature-level fusion outperforms all the single-modality classification algorithms in cognitive workload measurement, as indicated by its best and average accuracy. The best accuracy (93.21%) was obtained using ANN, which agrees with the research conducted by Movassagh et al. [54]. In their research, they revealed that ANN is more convergent with the neural network coefficient than the existing algorithms. Several studies followed a multimodal method to measure the cognitive load [19, 55, 56]. According to Novak et al., measuring the cognitive load with physiological signals and task performance features together can achieve higher accuracy than using physiological signals or task performance features individually [55]. Putze F et al. [57] combined skin conductance, EEG, respiration, and pulse to categorize CL into visual and cognitive tasks through simple majority voting fusion. The results show that decision-level fusion outperformed the single-modality method in one task, while it was surpassed in other tasks. According to Abdurrahman U. A. et al. [19], decision-level fusion outperforms feature-level fusion as well as single-modality methods with an accuracy of 94.67%. In another study conducted by Alzubi et al., a consensus-based combining method (CCM) was proposed and evaluated [58]. In thier study, the effectiveness of CCM was evaluated by comparing its performance with that of existing linear combination methods (majority voting, product, and average methods). The experimental results show that CCM provides a significant improvement in terms of accuracy over the product and average methods, in addition to demonstrating that the CCM’s classification accuracy is better than or comparable to that of majority voting.

Hussain S. et al. [59] combined galvanic skin response (GSR), ECG, Eye, and RESP features from physiological sensors into a classification model to investigate the cognitive load. Participants’ task performance features were applied to different classification models; sub-decisions were then combined using majority voting. The results show that hybrid-level fusion improved the classification accuracy by 6% compared to single classification methods. In another report by Abdurrahman U. A. et al., hybrid-level fusion performed better than feature-level and decision-level fusions with the highest accuracy, i.e., 97.14% [19].

## 5. Conclusions

This study investigated the effects of landmarks and routes on the navigational efficiency and learning transfer using a VR-based driving system. In addition, the fundamental reasons for these effects were thoroughly investigated. This study primarily aimed to measure both the psychophysiological and performance behaviors of the participants. Cognitive workload was applied using insufficient landmarks and difficult routes. The participants were required to use these landmarks to identify the correct directions to reach their destinations based on the knowledge acquired at the beginning of the exercise. While driving through these routes, driving performance and psychophysiological metrics were recorded simultaneously throughout the experiments. All the stated hypotheses of the study were confirmed by analyzing both the psychophysiological and performance features of the subjects. Human cognition and behavior correlate with psychophysiological characteristics that are strongly related to a constantly changing environment. The results of this study would help road administrators deduce how to correctly plan and accurately upgrade the operating conditions of public roads. It would also help them analyze traffic safety using driver cognition and driving performance data. A limitation of this study is that a driving simulator was used to collect data. However, data collected from the driving simulator can be easily controlled and reproduced, and dangerous driving conditions can be experienced without the risk of physical injury. Nevertheless, in the future, we will consider collecting data using real-world driving experiments and analyze the proposed hypotheses. The total number of participants in the study was 79. More samples may be required to obtain credible and robust results for a study of this nature. In the future, we will consider recruiting more participants to obtain more reliable and convincing results.
